The article "A Mathematical Model to Investigate the Transmission of COVID-19 in the Kingdom of Saudi Arabia" was published in 2020. Journal: Comput Math Methods Med.

# A Mathematical Model to Investigate the Transmission of COVID-19 in the Kingdom of Saudi Arabia

**DOI:** 10.1155/2020/9136157

**Published:** 2020-10-12

**Authors:** Fehaid Salem Alshammari

**Affiliations:** Department of Mathematics and Statistics, Imam Mohammad Ibn Saud Islamic University, Riyadh, Saudi Arabia

## Abstract

Since the first confirmed case of SARS-CoV-2 coronavirus (COVID-19) on March 02, 2020, Saudi Arabia has not reported quite a rapid COVD-19 spread as seen in America and many European countries. Possible causes include the spread of asymptomatic COVID-19 cases. To characterize the transmission of COVID-19 in Saudi Arabia, a susceptible, exposed, symptomatic, asymptomatic, hospitalized, and recovered dynamical model was formulated, and a basic analysis of the model is presented including model positivity, boundedness, and stability around the disease-free equilibrium. It is found that the model is locally and globally stable around the disease-free equilibrium when *R*_0_ < 1. The model parameterized from COVID-19 confirmed cases reported by the Ministry of Health in Saudi Arabia (MOH) from March 02 till April 14, while some parameters are estimated from the literature. The numerical simulation showed that the model predicted infected curve is in good agreement with the real data of COVID-19-infected cases. An analytical expression of the basic reproduction number *R*_0_ is obtained, and the numerical value is estimated as *R*_0_ ≈ 2.7.

## 1. Introduction

As of April 22, 2020, more than 12772 cases and 114 deaths of coronavirus disease 2019 (COVID-19) caused by the SARS-CoV-2 virus had been confirmed in the Kingdom of Saudi Arabia. Since March 04 [1], control measures have been implemented within Saudi Arabia to control the spread of the disease. Isolation of confirmed cases and contact tracing are crucial parts of these measures, which are common interventions for controlling infectious disease outbreaks [2–4]. For example, the severe acute respiratory syndrome (SARS) outbreak and the Middle East respiratory syndrome (MERS) were controlled through tracing suspected cases and isolating confirmed cases because the majority of transmission occurred concurrent or after symptom onset [3–5].

However, it is unknown if transmission of COVID-19 can occur before symptom onset, which could decrease the effectiveness of isolation and contact tracing [2, 3, 5].

In this paper, the impact of asymptomatic COVID-19 cases on the spread of the disease is considered using a modified version of the susceptible-exposed-infected-recovered (SEIR) dynamical model, along with the data of COVID-19 cases reported daily by the Ministry of Health in Saudi Arabia (MOH). Other main objectives of this paper include obtaining an analytical expression and numerical estimation of the basic reproduction number *R*_0_ of COVID-19 in Saudi Arabia and estimating the maximum required number of hospital beds and intensive care units (ICU). The rest of this study is organized as follows: The model establishment is presented in Section 2. Basic analysis of the model, including local and global stability results of the disease-free equilibrium, is explored in Section 3. The model fitting to daily reported cases and estimation of parameters is given in Section 4. Numerical results and discussion are presented in Section 5. Finally, brief concluding remarks are given in Section 6.

The article "A Mathematical Model to Investigate the Transmission of COVID-19 in the Kingdom of Saudi Arabia" was published in 2020. Journal: Comput Math Methods Med.

## 2. Model Establishment

The Saudi population *Q* will be divided into six categories: susceptible (*S*), exposed (*E*), symptomatic (*Y*), asymptomatic (*N*), hospitalized (*H*), and recovered (*R*) individuals (*SEYNHR*). Individuals move from the susceptible compartment *S* to the exposed compartment *E* after interacting with infected individuals with transmission rates *β*_1_, *β*_2_, and *β*_3_ as shown in Figure 1. COVID-19 is known to have an incubation period, from 2 to 14 days, between exposure and development of symptoms [6, 7]. After this period, exposed individual transits from the compartment *E* to either compartment *Y* at a rate *α* or compartment *N* at a rate *α*(1 − *γ*). An individual could move from compartment *N* to *Y* at a rate *K* if they show symptoms. Once an individual becomes infected with the coronavirus that causes COVID-19, that individual develops immunity against the virus with a rate *Φ*_*Y*_ or the individual will be hospitalized with a rate of *ε* or dies because of the disease with a rate of *μ*_1_. When an individual becomes hospitalized, that individual receives treatment and develops immunity against the virus with a rate *r* or dies because of the disease with a rate *μ*_2_.

As shown in Figure 1, the *SEYNHR* model has six compartments; therefore, a discrete dynamical system consisting of six nonlinear differential equations is formed as follows:

(1) $$\begin{array}{c} \frac{dS}{dt}=A-\left(\beta_{1}Y+\beta_{2}N+\beta_{3}H\right)S-\mu S, \end{array}$$

(2) $$\begin{array}{c} \frac{dE}{dt}=\left(\beta_{1}Y+\beta_{2}N+\beta_{3}H\right)S-\left(\alpha +\mu \right)E, \end{array}$$

(3) $$\begin{array}{c} \frac{dY}{dt}=\alpha \left(1-\gamma \right)E-\left(\Phi_{Y}+\varepsilon +\mu_{1}+\mu \right)Y+KN, \end{array}$$

(4) $$\begin{array}{c} \frac{dN}{dt}=\alpha \gamma E-\left(\Phi_{N}+K+\mu \right)N, \end{array}$$

(5) $$\begin{array}{c} \frac{dH}{dt}=\varepsilon Y-\left(r+\mu_{2}+\mu \right)H, \end{array}$$

(6) $$\begin{array}{c} \frac{dR}{dt}=\Phi_{Y}Y+\Phi_{N}N+rH-\mu R, \end{array}$$

where *Q*(*t*) = *S*(*t*) + *E*(*t*) + *Y*(*t*) + *N*(*t*) + *H*(*t*) + *R*(*t*) and *Q*(*t*) is the Saudi population at time *t*. The next-generation matrix is used in the next section to derive an analytical expression of the basic reproduction number *R*_0_, for the compartmental model above. Calculating *R*_0_ is a useful metric for assessing the transmission potential of an emerging COVID-19 in Saudi Arabia.

The article "A Mathematical Model to Investigate the Transmission of COVID-19 in the Kingdom of Saudi Arabia" was published in 2020. Journal: Comput Math Methods Med.

## 3. Basic Analytical Results

In this section, the positivity and boundedness of the proposed *SEYNHR* model solution (6) and stability of the model around the disease-free equilibrium is investigated. Furthermore, an analytical expression of the basic reproduction number *R*_0_ is established.

### 3.1. Positivity and Boundedness

To show that the *SEYNHR* model (6) is biologically well-behaved or epidemiologically meaningful, we must show that all its state variables are nonnegative and bounded for *t* > 0.

(7) $$\begin{array}{c} \frac{dS}{dt}=A-\left(\beta_{1}Y\left(t\right)+\beta_{2}N\left(t\right)+\beta_{3}H\left(t\right)\right)S\left(t\right)-\mu S\left(t\right). \end{array}$$

**Lemma 1 .**

For *t* > 0 and initial values *P*(0) ≥ 0, where *P*(*t*) = (*S*(*t*), *E*(*t*), *Y*(*t*), *N*(*t*), *H*(*t*), *R*(*t*)), the solution of the *SEYNHR* model (6) is nonnegative if they exist.

**Proof**

Assume *t*_1_ = {*t* > 0 : *P*(*t*) > 0 ∈ [0, *t*]}, then it follows from the first equation of (6) as

It can be written as

(8) $$\begin{array}{c} \frac{dS}{dt}\left\{S\left(t\right)\;\exp\left(\mu t+\int_{0}^{t}\left(\beta_{1}Y\left(\zeta \right)+\beta_{2}N\left(\zeta \right)+\beta_{3}H\left(\zeta \right)\right)S\left(\zeta \right)d\zeta \right)\right\}-A\;\exp\left(\mu t+\int_{0}^{t}\left(\beta_{1}Y\left(\zeta \right)+\beta_{2}N\left(\zeta \right)+\beta_{3}H\left(\zeta \right)\right)S\left(\zeta \right)d\zeta \right)=0. \end{array}$$

Hence,

(9) $$\begin{array}{c} S\left(t_{1}\right)\;\exp\left(\mu t_{1}+\int_{0}^{t_{1}}\left(\beta_{1}Y\left(\zeta \right)+\beta_{2}N\left(\zeta \right)+\beta_{3}H\left(\zeta \right)\right)S\left(\zeta \right)d\zeta \right)-S\left(0\right)=\int_{0}^{t_{1}}A\;\exp\left(\mu p+\int_{0}^{p}\left(\beta_{1}Y\left(\zeta \right)+\beta_{2}N\left(\zeta \right)+\beta_{3}H\left(\zeta \right)\right)S\left(\zeta \right)d\zeta \right)dp, \end{array}$$

which can be found as below

(10) $$\begin{array}{c} S\left(t_{1}\right)=S\left(0\right)\;\exp\left\{-\left(\mu t_{1}+\int_{0}^{t_{1}}\left(\beta_{1}Y\left(\zeta \right)+\beta_{2}N\left(\zeta \right)+\beta_{3}H\left(\zeta \right)\right)S\left(\zeta \right)d\zeta \right)\right\}+\exp\left\{-\left(\mu t_{1}+\int_{0}^{t_{1}}\left(\beta_{1}Y\left(\zeta \right)+\beta_{2}N\left(\zeta \right)+\beta_{3}H\left(\zeta \right)\right)S\left(\zeta \right)d\zeta \right)\right\}\times \int_{0}^{t_{1}}A\;\exp\left(\mu p+\int_{0}^{p}\left(\beta_{1}Y\left(\zeta \right)+\beta_{2}N\left(\zeta \right)+\beta_{3}H\left(\zeta \right)\right)S\left(\zeta \right)d\zeta \right)dp>0. \end{array}$$

Hence, *S*(*t*) is nonnegative for *t* > 0. In a similar way, it can be shown that *E* > 0, *Y* > 0, *N* > 0, *H* > 0, and *R* > 0 for *t* > 0.

(11) $$\begin{array}{c} \frac{dQ}{dt}=A-\mu Q\left(t\right)-\mu_{1}Y-\mu_{2}H\leq A-\mu Q\left(t\right). \end{array}$$

**Lemma 2 .**

*Ω* = {(*S*(*t*), *E*(*t*), *Y*(*t*), *N*(*t*), *H*(*t*), *R*(*t*)) ∈ *R*_+_^6^ ∪ {0}: 0 < *S*(*t*) + *E*(*t*) + *Y*(*t*) + *N*(*t*) + *H*(*t*) + *R*(*t*) ≤ *A*/*μ*} is the positively invariant region of the model (6) with nonnegative initial conditions in *R*_+_^6^.

The article "A Mathematical Model to Investigate the Transmission of COVID-19 in the Kingdom of Saudi Arabia" was published in 2020. Journal: Comput Math Methods Med.

**Proof**

Suppose *Q*(*t*) = *S*(*t*) + *E*(*t*) + *Y*(*t*) + *N*(*t*) + *H*(*t*) + *R*(*t*) holds for *t* ≥ 0, then we get

It is obvious that

(12) $$\begin{array}{c} Q\left(t\right)\leq Q\left(0\right)e^{-\mu t}+\frac{A}{\mu }\left(1-e^{-\mu t}\right). \end{array}$$

Thus, lim_*t*⟶∞_sup *Q*(*t*) ≤ *A*/*μ*. Furthermore, (*dQ*(*t*))/*dt* < 0 if *Q*(*t*) > *A*/*μ*. This shows that solutions of the model (6) point towards *Ω*. Hence, *Ω* is positively invariant and solutions of (6) are bounded.

### 3.2. Basic Reproduction Number *R*_0_

It can be easily verified that system (6) always has a disease-free equilibrium (DFE), which we will denote by *E*_0_, and it is given by

(13) $$\begin{array}{c} E_{0}=\left(\frac{A}{\mu },0,0,0,0,0\right). \end{array}$$

Next, we investigate an important concept in epidemiology which is the basic reproduction number, defined as “the expected number of secondary cases produced, in a completely susceptible population, by a typical infective individual” [8]. The next-generation method is used to calculate *R*_0_; more details about the method are in [8]. The system (6) can be rewritten as follows:

(14) $$\begin{array}{c} \frac{dw}{dt}=\Phi \left(w\right)-\Psi \left(w\right), \end{array}$$

where *F*≔(*F*1, *F*2, *F*3, *F*4, *F*5, *F*6)^*T*^ and *V*≔(*V*1, *V*2, *V*3, *V*4, *V*5, *V*6)^*T*^, or more explicitly

(15) $$\begin{array}{c} \left(\begin{array}{c} \dot{E}\\ \dot{Y}\\ \dot{N}\\ \dot{H}\\ \dot{R}\\ \dot{S} \end{array}\right)=\left(\begin{array}{c} \left(\beta_{1}Y+\beta_{2}N+\beta_{3}H\right)S\\ 0\\ 0\\ 0\\ 0\\ 0 \end{array}\right)-\left(\begin{array}{c} \left(\alpha +\mu \right)E\\ \left({}_{Y}+\varepsilon +\mu_{1}+\mu \right)Y-\alpha \left(1-\gamma \right)*E-KN\\ \left(\Phi_{N}+K+\mu \right)N-\alpha \gamma E\\ \left(r+\mu_{2}+\mu \right)H-\varepsilon Y\\ \left(P+\mu \right)R-\Phi_{Y}-\Phi_{N}-rH\\ \left(\beta_{1}Y+\beta_{2}N+\beta_{3}H\right)S-A-PR \end{array}\right). \end{array}$$

The Jacobian matrices of *F* and *V* evaluated at the solution *E*_0_^∗^ = (0, 0, 0, 0, 0, *A*/*μ*)^*T*^ are given by

(16) $$\begin{array}{c} {\left.F=\left({\frac{\partial \Phi_{i}}{\partial w_{j}}}_{E_{0}^{*}}\right)\right|}_{\begin{array}{c} 1\leq i,j\leq 4 \end{array}}=\left(\begin{array}{cccc} 0 & \frac{\beta_{1}A}{\mu } & \frac{\beta_{2}A}{\mu } & \frac{\beta_{3}A}{\mu }\\ 0 & 0 & 0 & 0\\ 0 & 0 & 0 & 0\\ 0 & 0 & 0 & 0 \end{array}\right),\\ {\left.V=\left({\frac{\partial \Psi_{i}}{\partial w_{j}}}_{\begin{array}{c} E_{0}^{*} \end{array}}\right)\right|}_{\begin{array}{c} 1\leq i,j\leq 4 \end{array}}=\left(\begin{array}{cccc} \alpha +\mu & 0 & 0 & 0\\ -\alpha \left(1-\gamma \right) & \Phi_{Y}+\varepsilon +\mu_{1}+\mu & -K & 0\\ -\alpha \gamma & 0 & \Phi_{N}+K+\mu & 0\\ 0 & -\varepsilon & 0 & r+\mu_{2}+\mu \end{array}\right). \end{array}$$

Direct calculations show that

(17) $$\begin{array}{c} V^{-1}=\left(\begin{array}{cccc} \frac{1}{\alpha +\mu } & 0 & 0 & 0\\ m_{1} & m_{4} & m_{6} & 0\\ m_{2} & 0 & m_{7} & 0\\ m_{3} & m_{5} & m_{8} & \frac{1}{r+\mu_{2}+\mu } \end{array}\right), \end{array}$$

where

(18) $$\begin{array}{c} \left\{\begin{array}{cc} m_{1}= & \frac{\alpha \left(1-\gamma \right)K+\alpha \left(1-\gamma \right)\mu +\alpha \left(1-\gamma \right)\Phi_{N}+K\alpha \gamma }{\left(\Phi_{Y}+\varepsilon +\mu_{1}+\mu \right)\left(\Phi_{N}+K+\mu \right)\left(\alpha +\mu \right)},\\ m_{2}= & \frac{\alpha \gamma }{\left(\alpha +\mu \right)\left(\Phi_{N}+K+\mu \right)},\\ m_{3}= & \frac{\varepsilon \left(\alpha \left(1-\gamma \right)K+\alpha \left(1-\gamma \right)\mu +\alpha \left(1-\gamma \right)\Phi_{N}+K\alpha \gamma \right)}{\left(\Phi_{Y}+\varepsilon +\mu_{1}+\mu \right)\left(\Phi_{N}+K+\mu \right)\left(\alpha +\mu \right)\left(r+\mu_{2}+\mu \right)},\\ m_{4}= & \frac{1}{\Phi_{Y}+\varepsilon +\mu_{1}+\mu },\\ m_{5}= & \frac{\varepsilon }{\left(\Phi_{Y}+\varepsilon +\mu_{1}+\mu \right)\left(r+\mu_{2}+\mu \right)},\\ m_{6}= & \frac{K}{\left(\Phi_{N}+K+\mu \right)\left(\Phi_{Y}+\varepsilon +\mu_{1}+\mu \right)},\\ m_{7}= & \frac{1}{\Phi_{N}+K+\mu },\\ m_{8}= & \frac{\varepsilon K}{\left(\Phi_{Y}+\varepsilon +\mu_{1}+\mu \right)\left(\Phi_{N}+K+\mu \right)\left(r+\mu_{2}+\mu \right)}. \end{array}\right. \end{array}$$

Denoting the 4 × 4 identity matrix by *ℐ*, the characteristic polynomial Γ(*λ*) of the matrix *FV*^−1^ is given by

(19) $$\begin{array}{c} \begin{array}{cc} \Gamma \left(\lambda \right) & =\det\left(FV^{-1}-\lambda I\right),\\ & =\frac{-\lambda^{3}\left(\left(\Phi_{N}+K+\mu \right)\left(\beta_{1}\mu +\left(r+\mu_{2}\right)\beta_{1}+\beta_{3}\varepsilon \right)A\alpha \left(1-\gamma \right)+\left(B_{1}+B_{2}\right)A\alpha \gamma \right)+\lambda^{4}}{\mu \left(\Phi_{Y}+\varepsilon +\mu_{1}+\mu \right)\left(\Phi_{N}+K+\mu \right)\left(\alpha +\mu \right)\left(r+\mu_{2}+\mu \right)}, \end{array} \end{array}$$

where

(20) $$\begin{array}{c} \left\{\begin{array}{c} B_{1}=\beta_{2}\mu^{2}+\left(\left(\mu_{1}+\mu_{2}+\Phi_{Y}+\varepsilon +r\right)\beta_{2}+\beta_{1}K\right)\mu +K\left(r+\mu_{2}\right)\beta_{1},\\ B_{2}=\left(r+\mu_{2}\right)\left(\Phi_{Y}+\varepsilon +\mu_{1}\right)\beta_{2}+\beta_{3}\varepsilon K. \end{array}\right. \end{array}$$

The solutions *λ*_1,2,3,4_ are given by

(21) $$\begin{array}{c} \left\{0,0,0,\frac{\left(\Phi_{N}+K+\mu \right)\left(\beta_{1}\mu +\left(r+\mu_{2}\right)\beta_{1}+\beta_{3}\varepsilon \right)A\alpha \left(1-\gamma \right)+\left(B_{1}+B_{2}\right)A\alpha \gamma }{\mu \left(\Phi_{Y}+\varepsilon +\mu_{1}+\mu \right)\left(\Phi_{N}+K+\mu \right)\left(\alpha +\mu \right)\left(r+\mu_{2}+\mu \right)}\right\}. \end{array}$$

Therefore, the reproduction number *R*_0_ for the *SEYNHR* model (6) is given by

(22) $$\begin{array}{c} R_{0}=\max\left\{\lambda_{1},\lambda_{2},\lambda_{3},\lambda_{4}\right\},=\frac{\left(\Phi_{N}+K+\mu \right)\left(\beta_{1}\mu +\left(r+\mu_{2}\right)\beta_{1}+\beta_{3}\varepsilon \right)A\alpha \left(1-\gamma \right)+\left(B_{1}+B_{2}\right)A\alpha \gamma }{\mu \left(\Phi_{Y}+\varepsilon +\mu_{1}+\mu \right)\left(\Phi_{N}+K+\mu \right)\left(\alpha +\mu \right)\left(r+\mu_{2}+\mu \right)}. \end{array}$$

For simplicity, let us denote

(23) $$\begin{array}{c} \rho_{1}=\alpha +\mu ,\\ \rho_{2}=\Phi_{Y}+\varepsilon +\mu_{1}+\mu ,\\ \rho_{3}=\Phi_{N}+K+\mu ,\\ \rho_{4}=r+\mu_{2}+\mu . \end{array}$$

In order to interpret the basic reproduction number *R*_0_, we split the above expression of *R*_0_ as follows:

(24) $$\begin{array}{c} R_{0}=R_{YH}+R_{EYNH1}+R_{EYNH2}, \end{array}$$

where

(25) $$\begin{array}{c} R_{YH}=\alpha \left(1-\gamma \right)\times \frac{A}{\mu }\times \frac{1}{\rho_{1}}\times \frac{1}{\rho_{1}\rho_{4}}\times \left(\beta_{1}\rho_{4}+\beta_{3}\varepsilon \right),\\ R_{EYNH1}=\alpha \gamma \times \frac{A}{\mu }\times \left(\frac{1}{\rho_{1}\rho_{2}\rho_{3}\rho_{4}}\times \beta_{3}\mu^{2}\frac{1}{\rho_{1}\rho_{2}\rho_{3}\rho_{4}}\times \beta_{1}K\left(r+\mu_{2}\right)+\frac{1}{\rho_{1}\rho_{2}\rho_{3}\rho_{4}}\times \left(\left(\mu_{1}+\mu_{2}+\Phi_{Y}+\varepsilon +r\right)\beta_{2}+\beta_{1}K\right)\mu \right),\\ R_{EYNH2}=\alpha \gamma \times \frac{A}{\mu }\left(\frac{1}{\rho_{1}\rho_{2}\rho_{3}\rho_{4}}\times \beta_{2}\left(r+\mu_{2}\right)\left(\rho_{2}-\mu \right)+\frac{1}{\rho_{1}\rho_{2}\rho_{3}\rho_{4}}\times \beta_{1}\varepsilon K\right). \end{array}$$

The first and second terms in *R*_*YH*_ show the probability of the total population becoming symptomatic upon infection multiplied by mean symptomatic, exposed, and hospitalized infectious periods multiplied by symptomatic and hospitalized contact rates. The first and second terms in *R*_*EYNH*1_ show the probability of the total population becoming asymptomatic multiplied by mean exposed, symptomatic, asymptomatic, and hospitalized infectious periods multiplied by symptomatic, asymptomatic, and hospitalized contact rates. Furthermore, the first and second terms in *R*_*EYNH*2_ show the probability of the total population becoming asymptomatic multiplied by mean exposed, symptomatic, asymptomatic, and hospitalized infectious periods multiplied by asymptomatic and hospitalized contact rates. The obtained analytical expression of *R*_0_ shows that asymptomatic as well as symptomatic cases of COVID-19 could drive the growth of the pandemic in Saudi Arabia.

The article "A Mathematical Model to Investigate the Transmission of COVID-19 in the Kingdom of Saudi Arabia" was published in 2020. Journal: Comput Math Methods Med.

### 3.3. Stability of Disease-Free Equilibrium

In this section, the local and global stability of the model (6) around the disease-free equilibrium is explored. The epidemiological implication of the local stability result of DFE is that a small influx of COVID-19 infection cases will not generate a COVID-19 outbreak if *R*_0_ < 1 while the global stability result of DFE indicates that any influx of COVID-19 infection cases will not generate a COVID-19 outbreak if *R*_0_ < 1.

(26) $$\begin{array}{c} J_{E_{0}}=\left(\begin{array}{cccccc} -\mu & 0 & -\frac{\beta_{1}A}{\mu } & -\frac{\beta_{2}A}{\mu } & -\frac{\beta_{3}A}{\mu } & 0\\ 0 & -\left(\alpha +\mu \right) & \frac{\beta_{1}A}{\mu } & \frac{\beta_{2}A}{\mu } & \frac{\beta_{3}A}{\mu } & 0\\ 0 & \alpha \left(1-\gamma \right) & -\left(\Phi_{Y}+\varepsilon +\mu_{1}+\mu \right) & K & 0 & 0\\ 0 & \alpha \gamma & 0 & -\left(\Phi_{N}+K+\mu \right) & 0 & 0\\ 0 & 0 & \varepsilon & 0 & -\left(r+\mu_{2}+\mu \right) & 0\\ 0 & 0 & \Phi_{Y} & \Phi_{N} & r & -\mu \end{array}\right). \end{array}$$

**Theorem 1 .**

The DFE *E*_0_ of the system (6) is locally asymptotically stable if *R*_0_ < 1 and unstable otherwise.

**Proof**

The Jacobian matrix *J*_*E*_0__ obtained at the DFE *E*_0_ is as follows:

Clearly, the eigenvalues −*μ* and −*μ* are negative real numbers. The remaining eigenvalues can be obtained through the following equation:

(27) $$\begin{array}{c} \lambda^{4}+C_{1}\lambda^{3}+C_{2}\lambda^{2}+C_{3}\lambda +C_{4}=0, \end{array}$$

where

(28) $$\begin{array}{c} \left\{\begin{array}{cc} C_{1}= & \Phi_{Y}+\Phi_{N}+K+4\mu +\alpha +\varepsilon +\mu_{1}+\mu_{2}+r,\\ C_{2}= & -\frac{A\alpha \beta_{1}\left(1-\gamma \right)}{\mu }+\beta_{1}\rho_{1}\rho_{2}\rho_{3}^{2}\rho_{4}\psi ,\\ C_{3}= & -\frac{\left(2A\beta_{1}\alpha +A\alpha \right)\left(1-\gamma \right)}{\mu }+\rho_{1}\rho_{2}\rho_{3}^{2}\rho_{4}\psi +2\beta_{1}\rho_{1}\rho_{2}\rho_{3}^{2}\rho_{4}\psi ,\\ C_{4}= & -\frac{\left(A\beta_{1}\alpha +A\alpha \right)\left(1-\gamma \right)}{\mu }+\rho_{1}\rho_{2}\rho_{3}^{2}\rho_{4}\psi +\beta_{1}\rho_{1}\rho_{2}\rho_{3}^{2}\rho_{4}\psi +\text{positive terms}, \end{array}\right. \end{array}$$

where *ψ* = (*β*_1_*μ* + (*r* + *μ*_2_)*β*_1_ + *β*_3_*ε*) and *C*_1_ is obviously positive. We can rewrite *R*_0_ as

(29) $$\begin{array}{c} R_{0}=\frac{A\alpha \left(1-\gamma \right)+\text{positive terms}}{\mu \rho_{1}\rho_{2}\rho_{3}^{2}\rho_{4}\psi }. \end{array}$$

Clearly if *R*_0_ < 1, then *C*_2_ is positive. Similarly, we can show that *C*_3_ and *C*_4_ are all positive if *R*_0_ < 1. Further, it is easy to show the remaining Routh-Hurtwiz condition for the fourth-order polynomial (27). Thus, the DFE is locally asymptotically stable if *R*_0_ < 1.

The article "A Mathematical Model to Investigate the Transmission of COVID-19 in the Kingdom of Saudi Arabia" was published in 2020. Journal: Comput Math Methods Med.

The global stability of DFE *E*_0_ of the COVID-19 transmission model is studied in the following result.

(30) $$\begin{array}{c} \Pi \left(t\right)=\frac{W_{1}}{Q}E+W_{2}Y+W_{3}N+W_{4}H, \end{array}$$

where *W*_*i*_ for *i* = 1, 2, 3, 4, are positive constants. Differentiating the function *Π*(*t*) with respect to *t* and using the solutions of system (6), we obtain

(31) $$\begin{array}{c} \frac{\Pi \left(t\right)}{dt}=W_{1}\left[\frac{\left(\beta_{1}Y+\beta_{2}N+\beta_{3}H\right)S}{Q}-\frac{\rho_{1}E}{Q}\right]+W_{2}\left[\alpha \left(1-\gamma \right)E-\rho_{2}Y+KY\right]+W_{3}\left[\alpha \gamma -\rho_{3}N\right]+W_{4}\left[\varepsilon Y-\rho_{4}H\right]\leq W_{1}\left[\left(\beta_{1}Y+\beta_{2}N+\beta_{3}H\right)-\rho_{1}E\right]+W_{2}\left[\alpha \left(1-\gamma \right)E-\rho_{2}Y+KY\right]+W_{3}\left[\alpha \gamma -\rho_{3}N\right]+W_{4}\left[\varepsilon Y-\rho_{4}H\right],\text{as }\frac{S+E}{Q}<1.=\left[W_{2}\alpha \left(1-\gamma \right)-\rho_{1}+W_{3}\alpha \gamma \right]E+\left[W_{1}\beta_{1}-W_{2}\rho_{2}+W_{4}\varepsilon \right]Y+\left[W_{1}\beta_{2}-W_{3}\rho_{3}\right]N+\left[W_{1}\beta_{3}-W_{4}\rho_{4}\right]H=\rho_{1}\left[\frac{W_{2}\alpha \left(1-\gamma \right)+W_{3}\alpha \gamma }{\rho_{1}}-1\right]E+\left[W_{1}\beta_{1}-W_{2}\rho_{2}+W_{4}\varepsilon \right]Y\rho_{1}\left[\frac{W_{2}\alpha \left(1-\gamma \right)+W_{3}\alpha \gamma }{\rho_{1}}-1\right]E+\left[W_{1}\beta_{1}-W_{2}\rho_{2}+W_{4}\varepsilon \right]Y+\left[W_{1}\beta_{2}-W_{3}\rho_{3}\right]N+\left[W_{1}\beta_{3}-W_{4}\rho_{4}\right]H \end{array}$$

**Theorem 2 .**

The article "A Mathematical Model to Investigate the Transmission of COVID-19 in the Kingdom of Saudi Arabia" was published in 2020. Journal: Comput Math Methods Med.

The DFE *E*_0_ of the system (6) is globally asymptotically stable if *R*_0_ < 1 and unstable otherwise.

**Proof**

Let us consider the following Lyapunov function, described in [9]:

Now choosing

(32) $$\begin{array}{c} W_{1}=1,\\ W_{2}=\frac{A\left[\beta_{1}\mu +\left(r+\mu_{2}\right)\beta_{1}+\beta_{3}\varepsilon \right]}{\mu \rho_{1}\rho_{2}\rho_{4}},\\ W_{3}=\frac{A\left(B_{1}+B_{2}\right)}{\mu \rho_{1}\rho_{2}\rho_{3}\rho_{4}},\\ W_{4}=1. \end{array}$$

We obtain

(33) $$\begin{array}{c} \frac{\Pi \left(t\right)}{dt}\leq \rho_{1}\left(R_{0}-1\right)E. \end{array}$$

Hence, if *R*_0_ < 1, then *Π*(*t*)/*dt* < 0. Therefore, the largest compact invariant set in *Ω* is the singleton set *E*_0_, and using LaSalle's invariant principle [10], *E*_0_ is globally asymptotically stable in *Ω*.

## 4. Model Fitting and Parameter Estimation

For the parameterizations of the model (6), we consider some of the parameter values from the literature and the rest are fitted to the data of daily total COVID-19 cases in Saudi Arabia from March 02, 2020, till April 14, 2020, using the nonlinear least square method implemented in MATLAB.

Considering the time unit to be days, we can estimate the following parameters:

- Natural death rate *μ*: the average life span of Saudi people is 74.87 years; therefore, we have *μ* = 1/(74.87 × 365) = 3.6593 × 10^−5^ per day [11]
- The birth rate *A* is obtained from *A*/*μ* = *Q*(0), where the total Saudi population *Q*(0) is 34218169; therefore, *A* = 1252 per day [11]

Mean asymptomatic infectious period *Φ*_*N*_ is assumed to be the same as the mean asymptomatic infectious period *Φ*_*Y*_ because there is no estimation available in the literature [5, 12]. The remaining system parameters are either estimated from literature or obtained using a nonlinear least-square curve fitting in MATLAB and given in Table 1. The basic steps in the parameter estimation procedure are described in [13, 14] and summarized as follows: system (6) can be expressed as

(34) $$\begin{array}{c} \frac{du}{dt}=Z\left(t,u,\theta \right),\;u\left(t_{0}\right)=u_{0}. \end{array}$$

The function *Z* is dependent on *t*, the vectors of the dependent variables *u*, and unknown parameters *θ* to be estimated. The least-square technique estimates the best values of the model parameters by minimizing the error between the reported data points ${\hat{y}}_{t_{i}}$ and the solution of the model *y*_*t*_*i*__ associated with the model parameters *θ*. The objective function used in the minimization procedure is given as *n* where it denotes the available real data points. To obtain the model parameters, we minimize the following objective function:

(35) $$\begin{array}{c} \hat{\theta }=\overset{n}{\underset{i=1}{\sum }}{\left(y_{t_{i}}-{\hat{y}}_{t_{i}}\right)}^{2}. \end{array}$$

(36) $$\begin{array}{c} \left\{\begin{array}{c} \min\hat{\theta }\\ s\text{ubject to equation }\left(4\right). \end{array}\right. \end{array}$$

The model (6) is solved using MATLAB solver *ode*45 which uses the Runge-Kutta methods to solve the initial value problem. Then, the *lsqcurvefit* package was implemented to fit model (6) to COVID-19 data of confirmed cases from March 02 till April 14, to estimate the parameters using the described approach above. In Figure 2 and Figure 3(a), the numerical simulation showed that the model predicted infected curve is in good agreement to the real data of infected cases.

The article "A Mathematical Model to Investigate the Transmission of COVID-19 in the Kingdom of Saudi Arabia" was published in 2020. Journal: Comput Math Methods Med.

## 5. Numerical Results and Discussion

To illustrate the numerical results, we take the initial population and subpopulations as *Q*(0) = 34218169, *Y*(0) = 2, *S*(0) = *Q*(0) − *Y*(0) = 34218167, and *E*(0) = *N*(0) = *H*(0) = *R*(0). The estimated values of parameters fitted from COVID-19 cases from March 02 till April 14 published by the Ministry of Health in Saudi Arabia (MOH) are presented in Table 1.  Figure 3 shows the simulation of the model (6) with parameter values in Table 1.  Figure 3(b) shows that about 18% of the entire Saudi population will be asymptomatic in the last week of May 2020, and about 17% will be exposed in the third week of May. The percentage of the entire population being symptomatic at any time will not exceed 1%, which is estimated to occur in the third week of May.

Moreover, as shown in Figure 3(c), about 60000 hospital beds and 18000 ICU beds are required (assuming 30% of the hospitalized cases need ICU [6]) immediately after the second week of May. As of April 2020, the Ministry of Health in Saudi Arabia designated 25 hospitals for COVID-19-infected patients with up to 80000 beds and 8000 intensive care unit (ICU) beds [15] and therefore extra 10000 ICU beds could be required.

The parameters *β*_1_, *β*_2_, and *β*_3_ represent the impact of effective contact on the disease transmission as shown in Figures 4, 5, and 6. The effective contact rate from asymptomatic to susceptible *β*_2_ has the greatest impact on the number of new COVID-19 symptomatic cases *Y*(*t*) as shown in Figure 5. This is because of the large number of asymptomatic cases in comparison to symptomatic cases in the same timescale as shown in Figure 3(b). Thus, social distancing (reduction of *β*_2_) is an effective strategy to control the spread of the disease. The effective contact rate from hospitalized to susceptible *β*_3_ has no impact on the number of new COVID-19 symptomatic cases *Y*(*t*) as shown in Figure 6 because of the small number of hospitalized cases in comparison to asymptomatic and symptomatic cases.  Figure 7 shows that increasing the rate of asymptomatic becomes symptomatic *K* decreases the number of new COVID-19 symptomatic cases *Y*(*t*) because decreasing *K* implies increasing the contact time between individuals with COVID-19 (with no treatment) and susceptible individuals.

The article "A Mathematical Model to Investigate the Transmission of COVID-19 in the Kingdom of Saudi Arabia" was published in 2020. Journal: Comput Math Methods Med.

Based on estimated and measured parameter values, the basic reproduction number is estimated as *R*_0_ ≈ 2.7. The variation of the basic reproduction number *R*_0_ for different values of *β*_1_ and *β*_2_ and *β*_1_ and *K* are shown in the heat maps in Figure 8. The upper heat map shows that decreasing the effective contact rate from symptomatic to susceptible *β*_1_ and the effective contact rate from asymptomatic to susceptible *β*_1_ will decrease the spread of the disease as *R*_0_ decreases and vice versa. The lower heat map of Figure 8 shows that increasing *K* increases *R*_0_ and vice versa. In reality, *R*_0_ is not a biological constant; it could fluctuate daily depending on environmental and social factors such as the percentage of the entire susceptible population wearing a suitable medical mask and practicing physical distancing. In the literature, estimates of *R*_0_ vary greatly: from 1 to 6 [13, 16–22] up to 26.5 [12]. This variation is because of the different assumptions and factors they had considered in their calculations.

Parameters with the highest degree of uncertainty are the effective contact rates from symptomatic to susceptible *β*_1_, from asymptomatic to susceptible *β*_2_, and from hospitalized to susceptible *β*_3_ (expected to be a fraction of *β*_1_ because of the protective measures in hospitals); the rate of asymptomatic becomes symptomatic *K* as well as the mean asymptomatic infectious period *Φ*_*N*_^−1^.

The maximum estimated value of *β*_1_ is 0.5 per day which is one half of the value reported by Li et al. [16]. This could be a reasonable estimation as we have not seen a similar scenario in Saudi Arabia after 5 weeks since reaching 100 confirmed cases on the 14th of March (week 7 since the first case) as we have seen in many other countries like China, America, and different European countries in the same timescale. This could be a result of the precautionary measures taken by the Saudi authorities, including the closure of schools and universities that started as early as March 08 (six days after the first confirmed COVID-19 case in Saudi Arabia).

## 6. Conclusion

The COVID-19 pandemic has rapidly spread out to most countries around the world. As of April 22, 2020, more than 12772 cases had been confirmed in Saudi Arabia alone. In this study, a mathematical model is formulated in order to study the transmission of COVID-19 in Saudi Arabia. Some basic properties of the model are presented in Section 3 including model positivity, boundedness, and local and global stability around the disease-free equilibrium. It is proven that the disease-free equilibrium is locally and globally stable when *R*_0_ < 1. The model parameterized from COVID-19 confirmed cases reported by the Ministry of Health in Saudi Arabia (MOH) from March 02 till April 14, while some parameters are estimated from the literature. The numerical simulation showed that the model predicted infected curve is in good agreement to the real data of infected cases. An analytical expression of the basic reproduction number *R*_0_ is obtained in Section 3, and the numerical value is estimated as *R*_0_ ≈ 2.7.

The article "A Mathematical Model to Investigate the Transmission of COVID-19 in the Kingdom of Saudi Arabia" was published in 2020. Journal: Comput Math Methods Med.

The contribution of undocumented COVID-19 infections (asymptomatic cases) on the transmission of the disease deserves further studies and investigations. The obtained analytical expression of *R*_0_, along with the numerical result in Figure 5, shows that asymptomatic transmission of COVID-19 could drive the growth of the pandemic in Saudi Arabia. Therefore, more testing and social distancing are needed to identify COVID-19 patients and to contain the spread of the disease.

## Figures and Tables

**Figure 1:** Schematic diagram of the *SEYNHR* compartment model. The arrows, except the black ones, represent a progression from one compartment to the next.

**Figure 2:** Data fitting to the reported cases in Saudi Arabia from March 02, 2020, till April 14, 2020, using model (6) and the nonlinear least-square method.

**Figure 3:** Numerical results of the *SEYNHR* model with the parameter listed in Table 1. (a) Shows the estimated number of symptomatic COVID-19 cases, with the published data by the Ministry of Health in Saudi Arabia of confirmed COVID-19 cases (blue circles). (b) Shows the estimated susceptible, exposed, symptomatic, asymptomatic, hospitalized, and recovered subpopulations. (c) Shows estimations of the hospitalized cases and the required ICU beds (black dashed line). The red line represents the number of hospital beds available, while the red dashed line represents the number of ICU beds available in Saudi Arabia.

**Figure 4:** Effective contact rate from symptomatic to susceptible *β*_1_ (a measure of social-distancing effectiveness) on the number of new COVID-19-infected cases *Y*(*t*). The baseline value of *β*_1_ is as given in Table 1.

**Figure 5:** Effective contact rate from asymptomatic to susceptible *β*_2_ (a measure of social-distancing effectiveness) on the number of new COVID-19-infected cases *Y*(*t*). The baseline value of *β*_2_ is as given in Table 1.

The article "A Mathematical Model to Investigate the Transmission of COVID-19 in the Kingdom of Saudi Arabia" was published in 2020. Journal: Comput Math Methods Med.

**Figure 6:** Effective contact rate from hospitalized to susceptible *β*_3_ on the number of new COVID-19-infected cases *Y*(*t*). The baseline value of *β*_3_ is as given in Table 1.

**Figure 7:** Impact of the rate of asymptomatic becomes symptomatic *K* on the number of new COVID-19-infected cases *Y*(*t*).

**Figure 8:** Heat maps showing the variation of *R*_0_ for different parameter values: the upper heat map shows the variation of *R*_0_ for different values for *β*_1_ and *β*_2_, and the lower heat map shows the variation of *R*_0_ for different values for *β*_1_ and *K*.

**Table 1:** Parameters used in the simulations.

Parameter	Description	Dimension	Value	A 95% confidence interval	Source
*N*	Population of Saudi Arabia in 2019.	Individual	34218169	—	[11]
*A*	Birth rate in Saudi Arabia in 2019.	Individual/day	1252	—	[11]
*μ*	Death rate in Saudi Arabia in 2019.	Day ^−1^	3.6593x10^−5^	—	[11]
*β*_1_	Effective contact rate from symptomatic to susceptible.	Day ^−1^	0.35	[0.267, 0.5]	Fitted
*β*_2_	Effective contact rate from asymptomatic to susceptible.	Day ^−1^	0.7	[0.53, 1]	Fitted
*β*_3_	Effective contact rate from hospitalized to susceptible.	Day ^−1^	0.18	[0.13, 0.26]	Fitted
*α* ^−1^	Mean latent period.	Days	5.1	—	[23]
*γ*	Probability of becoming asymptomatic upon infection.	n/a	0.86	—	[24]
*Φ*_*Y*_^−1^	Mean symptomatic infectious period.	Days	8	—	[25]
*ε*	Rate of symptomatic becomes hospitalized.	Day ^−1^	0.125	—	[1]
*μ*_1_	Death rate of symptomatic patients.	Day ^−1^	0.392	—	[26]
*K*	Rate of asymptomatic becomes symptomatic.	Day ^−1^	0.12	[0.1, 0.125]	Fitted
*Φ*_*N*_^−1^	Mean asymptomatic infectious period.	Days	8	—	Assumed
*r*	Rate of recovered hospitalized patients.	Day ^−1^	0.1	—	[6]
*μ*_2_	Death rate of hospitalized patients.	Day ^−1^	0.392	—	[1]

## Data Availability

The data used in my paper is the total number of confirmed cases of COVID-19 reported by the Ministry of Health in Saudi Arabia from the 2nd of March until the 21st of April 2020. Data supporting this paper are open and can be accessed through (in Arabic) Ministry of Health COVID 19 Dashboard. Saudi Arabia; 2020 (https://covid19.moh.gov.sa). Alternatively, data supporting this paper are open and can be accessed through (in English) Our World in Data; Oxford; 2020 (https://covid.ourworldindata.org/data/owid-covid-data.csv).
